The article "Dynamic Harmony Search with Polynomial Mutation Algorithm for Valve-Point Economic Load Dispatch" was retracted in 2016. Reason: concerns about the peer review.

# Dynamic Harmony Search with Polynomial Mutation Algorithm for Valve-Point Economic Load Dispatch

**DOI:** 10.1155/2015/147678

**Published:** 2015-09-30

**Authors:** M. Karthikeyan, T. Sree Ranga Raja

**Affiliations:** ^1^Department of Electrical and Electronics Engineering, University College of Engineering Pattukkottai, Rajamadam, Tamilnadu 614701, India; ^2^Department of Electrical and Electronics Engineering, University College of Engineering, Nagerkovil, Tamilnadu 629001, India

## Abstract

Economic load dispatch (ELD) problem is an important issue in the operation and control of modern control system. The ELD problem is complex and nonlinear with equality and inequality constraints which makes it hard to be efficiently solved. This paper presents a new modification of harmony search (HS) algorithm named as dynamic harmony search with polynomial mutation (DHSPM) algorithm to solve ORPD problem. In DHSPM algorithm the key parameters of HS algorithm like harmony memory considering rate (HMCR) and pitch adjusting rate (PAR) are changed dynamically and there is no need to predefine these parameters. Additionally polynomial mutation is inserted in the updating step of HS algorithm to favor exploration and exploitation of the search space. The DHSPM algorithm is tested with three power system cases consisting of 3, 13, and 40 thermal units. The computational results show that the DHSPM algorithm is more effective in finding better solutions than other computational intelligence based methods.

## 1. Introduction

Economic load dispatch (ELD) is an important issue in the operation and control of modern control system. The objective of ELD problem can be defined as determining the real power outputs of generators so as to meet the required load demand at minimum operating cost while satisfying system equality and inequality constraints [1]. The objective of ELD is to minimize the total operating cost, but the various types of physical and operational constraints make ELD a highly nonlinear constrained optimization problem. Traditionally different approaches have been suggested to solve ELD, including linear programming [2], dynamic programming [3], and nonlinear programming [4]. The main drawback of these techniques is that they may not be able to give an optimal solution and may get stuck at local optima.

Recently, different heuristic approaches have been used to solve ELD problem with promising performance, such as genetic algorithm (GA) [5], evolutionary programming (EP) [6], differential evolution (DE) [7], and particle swarm optimization (PSO) [8]. In spite of the fact that these heuristic methods do not always guarantee finding global optimal solutions in specified time, they often provide fast and reasonable solution. Although several heuristic methodologies have been developed for the ELD problem, the difficulty of the problem reveals the need for development of efficient algorithms to exactly locate the optimum solution.

The article "Dynamic Harmony Search with Polynomial Mutation Algorithm for Valve-Point Economic Load Dispatch" was retracted in 2016. Reason: concerns about the peer review.

Harmony search (HS) is a new metaheuristic algorithm proposed by Geem et al. [9], which is inspired by the natural musical performance process that happens when a musician searches for a better state of harmony. HS algorithm has been successfully applied to a wide range of applications such as structural optimization [10], design optimization of water distribution networks [11], and vehicle routing [12].

Although HS algorithm is good at identifying the solution in the search space within a reasonable time, it is not efficient in performing local search in numerical optimization applications [13]. To overcome this drawback, Mahdavi et al. [13] proposed an improved HS algorithm denoted as improved harmony search (IHS) by dynamically updating pitch adjustment rate (PAR) and bandwidth (bw). Omran and Mahdavi [14] proposed a global best HS algorithm denoted as global harmony search (GHS) by borrowing the idea from swarm intelligence. Khalili et al. [15] proposed global dynamic harmony search (GDHS) algorithm for solving continuous optimization problem.

In this paper, we present a novel variant of HS algorithm, named dynamic harmony search with polynomial mutation (DHSPM) algorithm in which harmony memory considering rate (HMCR) and pitch adjusting rate (PAR) are dynamically updated. Additionally, polynomial mutation is inserted in the updating step of HS algorithm to favor exploration and exploitation of the search space.

The paper is organized as follows.  Section 2 presents the formulation of ELD problem with valve-point.  Section 3 contains a brief overview of HS and DHSPM algorithms.  Section 4 reports the application of DHSPM to ELD problem with valve-point effect.  Section 5 contains the description of the simulations and a discussion of the results. Conclusions are summarized in Section 6.

## 2. Problem Formulation

### 2.1. Economic Dispatch

The primary objective of the ELD problem is to determine the most economic loading of the generators such that the total demand is met while satisfying equality and inequality constraints. The objective function of ELD is defined as

(1) $$\begin{array}{c} \min F_{T}=\min\overset{N}{\underset{i=1}{\sum }}F_{i}\left(\;P_{i}\;\right). \end{array}$$

*F*_*T*_ is the objective function describing the total generation cost. *F*_*i*_(*P*_*i*_) is the cost function of generator *i* to generate real power *P*_*i*_. *N* is the total number of generators in the power system.

The article "Dynamic Harmony Search with Polynomial Mutation Algorithm for Valve-Point Economic Load Dispatch" was retracted in 2016. Reason: concerns about the peer review.

The fuel cost function of unit *i* is defined by

(2) $$\begin{array}{c} F_{i}\left(\;P_{i}\;\right)=a_{i}P_{i}^{2}+b_{i}P_{i}+c_{i}, \end{array}$$

where *a*_*i*_, *b*_*i*_, and *c*_*i*_ are the cost coefficients of unit *i*.

### 2.2. Economic Load Dispatch with Valve-Point Loading Effects

Multivalve steam turbines based generating units are characterized by complex nonlinear fuel cost function. This is mostly due to the ripples made by the valve-point loading. To simulate these complex phenomena, a sinusoidal component is added on the quadratic heat rate curve. To take into account this effect, the cost function in (2) is modified as follows:

(3) $$\begin{array}{c} F_{i}\left(\;P_{i}\;\right)=a_{i}+b_{i}P_{i}+c_{i}P_{i}^{2}+\left|\;e_{i}\sin\left(\;f_{i}\left(\;P_{i}^{\min}-P_{i}\;\right)\;\right)\;\right|, \end{array}$$

where *e*_*i*_ and *f*_*i*_ denote the cost coefficients of *i*th generator reflecting valve-point loading effect and *P*_*i*_^min⁡^ is the minimum output power of *i*th generator unit.

### 2.3. Constraints

#### 2.3.1. Real Power Balance Constraint

The total power generated should be equal to the total load demand plus the total transmission losses. The real power balance can be expressed as

(4) $$\begin{array}{c} \overset{N}{\underset{i=1}{\sum }}P_{i}=P_{D}+P_{L}, \end{array}$$

where *P*_*D*_ is the total demand and *P*_*L*_ denotes the total transmission losses. In this paper, we disregarded the transmission loss, *P*_*L*_ = 0.

#### 2.3.2. Generator Capacity Constraints

Real power output of each generator should be within its minimum and maximum limits. This can defined as follows:

(5) $$\begin{array}{c} P_{i,\min}\leq P_{i}\leq P_{i,\max}, \end{array}$$

where *P*_*i*,min⁡_ and *P*_*i*,max⁡_ are the minimum and maximum output power of *i*th generating unit, respectively.

### 2.4. Formulation of Fitness Function

In this paper, we use penalty term to transform a constrained optimization problem into an unconstrained one. As a result, the fitness function can be written as

(6) $$\begin{array}{c} \mathrm{Min}F=\overset{n}{\underset{i=1}{\sum }}F_{i}\left(\;P_{i}\;\right)+\gamma \left|\;\overset{n}{\underset{i=1}{\sum }}P_{i}-\left(\;P_{D}+P_{L}\;\right)\;\right|, \end{array}$$

where *γ* is the penalty coefficient. The penalty coefficient should be given large enough to guarantee the system constraints. In this paper, we choose *γ* = 1000.

## 3. Harmony Search Algorithms

### 3.1. Basic Harmony Search Algorithm

In basic harmony search (HS) algorithm, each solution is called a “harmony” and represented by an *n*-dimensional real vector. An initial population of harmony vectors is randomly created to form a harmony memory (HM). Then, a new harmony vector is generated by using a memory consideration rule, a pitch adjustment rule, and a random reinitialization. The generated new harmony vector is updated in the HM by comparing the new harmony vector and the worst harmony vector in the HM. The above process is repeated until a certain criterion is met. The steps of HS algorithm are described below in detail.

The article "Dynamic Harmony Search with Polynomial Mutation Algorithm for Valve-Point Economic Load Dispatch" was retracted in 2016. Reason: concerns about the peer review.

**Step 1 (initialization of problem and algorithm parameters).**

Consider an optimization problem that is described by

(7) $$\begin{array}{c} \text{Minimize}\;F\left(\;x\;\right)\;x_{i}\in X_{i},\;\;i=1,2,\ldots ,N, \end{array}$$

where *F*(*x*) is the objective function, *x* is the set of design variables, and *X*_*i*_ is the range set of the possible values for each design variable. The parameters of the HS algorithm are the harmony memory size (HMS), harmony memory considering rate (HMCR), pitch adjusting rate (PAR), number of decision variables (*N*), and number of improvisations (NI).

**Step 2 (harmony memory initialization).**

The harmony memory (HM) matrix is filled with randomly generated solution vectors for HMS and sorted by the values of objective function *f*(*x*) as shown below:

(8) HM=x11x21⋯xN−11xN1x12x22⋯xN−12xN2⋮⋮⋯⋮⋮x1HMS−1x2HMS−1⋯xN−1HMS−1xNHMS−1x1HMSx2HMS⋯xN−1HMSxNHMS⟶fx1⟶fx2⋮⟶fxHMS−1⟶fxHMS.

**Step 3 (new harmony improvisations).**

A new harmony vector *X*_new_ is created by applying three rules: a memory consideration, a pitch adjustment, and a random selection. A random number *r*_1_ between 0 and 1 is generated. If *r*_1_ is less than HMCR, then *X*_new_ is generated by the memory consideration; otherwise, *X*_new_ is obtained by randomly generating a vector between the upper and lower bounds. In the memory consideration, *X*_new_ is selected from any harmony vector in HM. After memory consideration, *X*_new_ will undergo a pitch adjustment with a probability of PAR. The pitch adjustment rule is given as follows:

(9) $$\begin{array}{c} X_{\text{new}}=X_{\text{new}}\pm r\times \text{bw}, \end{array}$$

where *r* is a random number generated between 0 and 1.

**Step 4 (updating harmony memory).**

If the new harmony vector *X*_new_ has better fitness function than the worst harmony in the HM, the new harmony is included in the HM and the existing worst harmony is excluded from the HM.

**Step 5 (checking the stopping criterion).**

If the stopping criterion, which is based on the maximum number of improvisations, is satisfied, the computation is terminated. Otherwise, Steps 3 and 4 are repeated.

### 3.2. Variants of HS Algorithm

Mahdavi et al. proposed improved harmony search (IHS) algorithm to address the limitations of the basic HS algorithm. IHS algorithm applies the same memory consideration, pitch adjustment, and random selection as the basic HS algorithm, but the author suggests a new formula for PAR and bw which dynamically changes at every iteration [13].

The article "Dynamic Harmony Search with Polynomial Mutation Algorithm for Valve-Point Economic Load Dispatch" was retracted in 2016. Reason: concerns about the peer review.

Omran and Mahdavi proposed a global best harmony search (GHS) algorithm which is based on the inspiration by the particle swarm optimization. Unlike the basic HS algorithm, the GHS algorithm generates a new harmony vector by making use of the best harmony vector [14].

Khalili et al. proposed a global dynamic harmony search (GDHS) algorithm by modifying the basic HS algorithm to solve continuous optimization problems [15].

Pan et al. proposed a self-adaptive global best harmony (SGHS) algorithm for solving continuous optimization problem. In SGHS, new improvisation scheme was suggested so that good information obtained in the current global best solution is utilized to generate new harmonies [16].

### 3.3. Dynamic Harmony Search with Polynomial Mutation (DHSPM) Algorithm

In this paper, a novel HS algorithm, called DHSPM, for solving ORPD problem of power system, is presented. The proposed algorithm is different from the classical HS algorithm in the following two aspects. First, a dynamic parameter adjustment scheme is suggested, which can dynamically update the parameters HMCR and PAR in every improvisation. Second, a polynomial mutation is inserted in the updating step of HS algorithm to favor exploration and exploitation of the search space. The details of the algorithm are given below.

#### 3.3.1. Dynamic Control Parameters

The conventional HS algorithm uses fixed value for both HMCR and PAR. In the HS algorithm, HMCR and PAR are fixed in the initialization step and cannot be changed during the improvisation. The main drawback of this method is that the number of iterations needed to find optimal solution is more [13]. Here, we suggest dynamic formula for HMCR and PAR which change during the improvisation of the optimization. The suggested formulas for HMCR and PAR for the current improvisation *t* are

(10) HMCRC1∗t+0.90≤t≤NI2−C1∗t+1.1NI2≤t≤NI,PAR=C2∗t+0.30≤t≤NI2−C2∗t+1.1NI2≤t≤NI,

where

(11) C11−0.9NI/2,C2=0.7−0.3NI/2.

Figures 1 and 2 show the schematic of HMCR and PAR in dynamic mode for the number of improvisations equal to 1000. At initial improvisations, a linear increase of HMCR makes the algorithm generate more new harmony vectors rather than choosing from the harmony memory. At the middle of the improvisations, the HMCR is equal to 1, which consider the harmony vector from the HM itself. At final improvisations, HMCR is linearly decreased, which helps to escape the optimization process from settling in local optima. Similarly, the large value of PAR at the middle of the improvisation enforces the selected harmony vector to have adjustments.

The article "Dynamic Harmony Search with Polynomial Mutation Algorithm for Valve-Point Economic Load Dispatch" was retracted in 2016. Reason: concerns about the peer review.

#### 3.3.2. Polynomial Mutation

Mutation is an important operator in genetic algorithms (GAs), as it ensures the maintenance of diversity in the evolving populations of GAs [17]. There are several mutation techniques that can be used in genetic algorithms like random mutation [18], boundary mutation [18], nonuniform random mutation [19], power mutation [17], polynomial mutation [18], and so forth. The experimental evaluation of the HS algorithm using different mutation methods using a well-known set of test functions shows that using the polynomial mutation improves the performance of the algorithm significantly for a considerable number of functions [20]. Deb and Agrawal [18] suggested a polynomial mutation operator with a user-defined index parameter (*η*_*m*_). They concluded that *η*_*m*_ induces an effect of a perturbation of *O*((*b* − *a*)/*η*_*m*_) in a variable, where *a* and *b* are lower and upper bounds. They also found that a value *η*_*m*_ ∈ [20, 100]  is adequate in most problems that they tried of the variable. In this paper, we suggest inserting polynomial mutation in the updating step of HS algorithm as follows:

(12) xnew′j=xnewj+δ1xnewj−xlower,jfor  r≤0.5xnewj+δ2xupper,j−xnewjfor  r>0.5.

Then, either of the two parameters (*δ*_1_ or *δ*_2_) is calculated as follows:

(13) δ12r1/1+ηm−1for  r≤0.5,δ2=1−21−r1/1+ηmfor  r>0.5,

where *x*_new_(*j*) is the new harmony vector selected at the updating step of HS algorithm,  *x*_new_′(*j*) is the mutated new harmony vector, and *r* is a random number created within [0,1].

The optimization procedure of DHSPM is as follows.

**Step 1 .**

Set the parameters HMS, bw, and NI.

**Step 2 .**

Initialize the HM and calculate the objective function of each harmony vector.

**Step 3 .**

Determine new harmony vector *x*_new_(*j*) as follows:

 for (*j* = 1 : *N*), do
  (14) HMCRC1∗t+0.90≤t≤NI2−C1∗t+1.1NI2≤t≤NI,PAR=C2∗t+0.30≤t≤NI2−C2∗t+1.1NI2≤t≤NI,C1=1−0.9NI/2,C2=0.7−0.3NI/2
 if (*r*_1_ < HMCR) then
  (15) $$\begin{array}{c} x_{\text{new}}\left(\;j\;\right)=x_{a}\left(\;j\;\right)\;a\in \left(1,2,\ldots ,\text{HMS}\right) \end{array}$$
 if (*r*_2_ < PAR) then
  (16) $$\begin{array}{c} x_{\text{new}}\left(\;j\;\right)=x_{\text{new}}\left(\;j\;\right)\pm \text{bw}\;r_{1},r_{2}\in \left(0,1\right) \end{array}$$
 endif
 else
  (17) xnewj=xlower,j+r3×xupper,j−xlower,jr3∈0,1
 endif
 endfor

**Step 4 (updating of HM).**

If the new harmony vector *x*_new_(*j*) is better than the worst harmony in HM, the mutated new harmony vector *x*_new_′(*j*)  is created as follows:

(18) xnew′j=xnewj+δ1xnewj−xlower,jfor  r≤0.5xnewj+δ2xupper,j−xnewjfor  r>0.5,δ1=2r1/1+ηm−1for  r≤0.5,δ2=1−21−r1/1+ηmfor  r>0.5.

The article "Dynamic Harmony Search with Polynomial Mutation Algorithm for Valve-Point Economic Load Dispatch" was retracted in 2016. Reason: concerns about the peer review.

The mutated new harmony vector *x*_new_′(*j*) is inserted into the HM, and the worst harmony is removed from the HM.

**Step 5 .**

If maximum number of improvisations (NI) is reached, the computation is terminated. Otherwise, Steps 3 and 4 are repeated.

#### 3.3.3. Study on Benchmark Functions

To test the performance of the proposed DHSPM algorithm, an extensive experimental evaluation is provided based on a set of 7 global optimization problems as follows.

*Sphere Function *(*f*_1_). Sphere function is defined as

(19) $$\begin{array}{c} \min f\left(\;x\;\right)=\overset{n}{\underset{i=1}{\sum }}x^{2}\left(\;i\;\right), \end{array}$$

where global optimum *x* ^∗^ = 0 and *f*(*x* ^∗^) = 0 for −100 ≤ *x*(*i*) ≤ 100.

*Schwefel's Problem 2.22 *(*f*_2_). Schwefel's problem 2.22 is defined as

(20) $$\begin{array}{c} \min f\left(\;x\;\right)=\overset{n}{\underset{i=1}{\sum }}\left|\;x\left(\;i\;\right)\;\right|+\overset{n}{\underset{i=1}{\prod }}\left|\;x\left(\;i\;\right)\;\right|, \end{array}$$

where global optimum *x* ^∗^ = 0 and *f*(*x* ^∗^) = 0 for −10 ≤ *x*(*i*) ≤ 10. 

*Rosenbrock Function *(*f*_3_). Rosenbrock function is defined as

(21) min⁡⁡fx=∑i=1n−1100xi+1−x2i2+xi−12,

where global optimum *x* ^∗^ = (1,1,…, 1) and *f*(*x* ^∗^) = 0 for −30 ≤ *x*(*i*) ≤ 30.

*Step Function *(*f*_4_). Step function is defined as

(22) $$\begin{array}{c} \min f\left(\;x\;\right)=\overset{n}{\underset{i=1}{\sum }}{\left(\;\left|\;x\left(i\right)+0.5\;\right|\;\right)}^{2}, \end{array}$$

where global optimum *x* ^∗^ = 0 and *f*(*x* ^∗^) = 0 for −100 ≤ *x*(*i*) ≤ 100. 

*Rotated Hyperellipsoid Function *(*f*_5_). Rotated hyperellipsoid function is defined as

(23) $$\begin{array}{c} \min f\left(\;x\;\right)=\overset{n}{\underset{i=1}{\sum }}{\left(\;\overset{i}{\underset{j=1}{\sum }}x\left(\;j\;\right)\;\right)}^{2}, \end{array}$$

where global optimum *x* ^∗^ = 0 and *f*(*x* ^∗^) = 0 for −100 ≤ *x*(*i*) ≤ 100. 

*Schwefel's Problem 2.26 *(*f*_6_). Schwefel's problem 2.26 is defined as

(24) $$\begin{array}{c} \min f\left(\;x\;\right)=418.9829n-\overset{n}{\underset{i=1}{\sum }}\left(\;x\left(\;i\;\right)\sin\left(\;\sqrt{\left|x\left(i\right)\right|}\;\right)\;\right), \end{array}$$

where global optimum *x* ^∗^ = (420.9687,420.9687,…, 420.9687) and *f*(*x* ^∗^) = 0 for −500 ≤ *x*(*i*) ≤ 500. 

*Rastrigin Function *(*f*_7_). Rastrigin function is defined as

(25) $$\begin{array}{c} \min f\left(\;x\;\right)=\overset{n}{\underset{i=1}{\sum }}\left(\;x^{2}\left(\;i\;\right)-10\cos\left(\;2\pi x\left(i\right)\;\right)+10\;\right), \end{array}$$

where global optimum *x* ^∗^ = 0 and *f*(*x* ^∗^) = 0 for −5.12 ≤ *x*(*i*) ≤ 5.12.

The article "Dynamic Harmony Search with Polynomial Mutation Algorithm for Valve-Point Economic Load Dispatch" was retracted in 2016. Reason: concerns about the peer review.

The parameters of DHSPM are HM = 5, bw = 0.01, and *η*_*m*_ = 10. Thirty independent replications are carried out for each function and the number of improvisations (NI) for each run is set to 10000. The average and standard deviations (SD) generated by the three algorithms (HS, IHS, and DHSPM) with dimension 30 are reported in Table 1. It can be seen from Table 1 that DHSPM generates best results for 7 functions compared to HS and IHS algorithms.

## 4. Application of DHSPM for ELD Problem

In this section, the DHSPM algorithm is applied for economic load dispatch problem with valve-point effect. The main steps symbolizing the search procedure are given below.

**Step 1 .**

Specify the generator cost coefficients and valve-point coefficients, choose the number of generator units (*N*), and specify maximum and minimum real power generation capacity of all generators and load demand *P*_*D*_. Initialize the parameters of DHSPM.

**Step 2 .**

Initialize HM matrix with size HMS × *N*, where *N* represents the total number of generators in the system.

**Step 3 .**

Calculate the fitness value for each harmony vector in the HM using (6). The penalty factors are chosen high enough to make constraint violations prohibitive in the final solution. Use penalty coefficient *γ* = 1000.

**Step 4 .**

Calculate HMCR and PAR using (10).

**Step 5 .**

Generate new harmony vector using random selection, memory consideration, and pitch adjustment.

**Step 6 .**

If the new harmony vector is better than the worst harmony in the HM, then calculate the mutated new harmony using (12) and include it in HM.

**Step 7 .**

If the maximum number of improvisations is reached, go to Step 8; otherwise, repeat Steps 4–6.

**Step 8 .**

Print the optimal value of real power generation of generators and total cost of generation.

## 5. Simulation and Results

In this section, the DHSPM algorithm was tested with three standard load dispatch problems (3, 13, and 40 thermal units). The software was written in MATLAB 2009b and applied on a 2.40 GHz Intel Core i5 CPU personal computer with 4 GB RAM. The parameters of DHSPM for all the test systems are given in Table 2

### 5.1. 3 Thermal Units

A system of three thermal units with the valve-point loading was considered in this test. In this case, the load demand is taken as *P*_*D*_ = 850 MW. The test system comprises three generating units with quadratic cost functions together with the effects of valve-point loadings as given in Table 3. Based on data attained through 100 trials, the comparisons of the three thermal units test by different algorithm are represented in Tables 4 and 5, which show that the DHSPM also succeeded in finding the satisfactory solution. The fuel cost convergence of harmony search algorithms for 3 thermal units is shown in Figure 3.

The article "Dynamic Harmony Search with Polynomial Mutation Algorithm for Valve-Point Economic Load Dispatch" was retracted in 2016. Reason: concerns about the peer review.

### 5.2. 13 Thermal Units

A system of 13 generating units with the valve-point loadings is given in Table 6. In this case, the load demand is considered as *P*_*D*_ = 1800 MW. The optimal real power generation outputs of 13 generators using DHSPM after conducting 100 trails is given in Table 7. The comparisons of the 13 thermal units test by different methods with DHSPM obtained through 100 trials are given in Table 8. From Table 8, it can be observed that the DHSPM algorithm succeeds in finding a satisfactory solution. Table 8 also summarizes the minimum and average cost obtained by all algorithms. From Table 8, the minimum cost obtained by DHSPM is 17960.54 $/h which is the best cost found so far. The fuel cost convergence of harmony search algorithms for 13 thermal units is shown in Figure 4.

### 5.3. 40 Thermal Units

In order to test DHSPM algorithm deeper, a system of 40 thermal units with the effects of valve-point loading was considered in this test. The data of 40 thermal units with valve-point loading effect is given in Table 9. In this case, the load demand is equal to *P*_*D*_ = 10500 MW. The optimal value of real power generation by DHSPM after conducting 100 trails is depicted in Table 10. The results obtained by applying the DHSPM algorithm and other algorithms are summarized in Table 11. From Table 11, it can be concluded that the DHSPM method succeeds in finding a satisfactory solution. Table 11 also summarizes the minimum and average cost obtained by other settled algorithms. From Table 11, the minimum cost obtained by DHSPM is 121412.66 $/h which is the best cost when compared with other existing algorithms. The fuel cost convergence of harmony search algorithms for 40 thermal units is shown in Figure 5.

## 6. Conclusion

In this paper, dynamic harmony search with polynomial mutation algorithm is applied to solve economic load dispatch problem with valve-point loading effect. The feasibility and the effectiveness of DHSPM algorithm have been investigated on three test systems having 3, 13, and 40 units. The DHSPM algorithm achieves the minimum fuel cost for the above unit cases when compared with other optimization methods reported in the literature. The successful optimizing performance on the validation data sets proves the efficiency of the DHSPM algorithm and shows that it can be used as a reliable tool for economic load dispatch problem.

## Figures and Tables

**Figure 1:** Variations of HMCR with respect to improvisations.

The article "Dynamic Harmony Search with Polynomial Mutation Algorithm for Valve-Point Economic Load Dispatch" was retracted in 2016. Reason: concerns about the peer review.

**Figure 2:** Variations of PAR with respect to improvisations.

**Figure 3:** Fuel cost convergence nature of DHSPM, IHS, and HS for 3 thermal units' system.

**Figure 4:** Fuel cost convergence nature of DHSPM, IHS, and HS for 13 thermal units' system.

**Figure 5:** Fuel cost convergence nature of DHSPM, IHS, and HS for 40 thermal units' system.

**Table 1:** Mean and standard deviation of the benchmark functions.

Function	HS	IHS	DHSPM
*f*_1_	7.711433 (3.307032)	0.000000 (0.000000)	0.000000 (0.000000)
*f*_2_	0.112437 (0.059248)	0.000009 (0.000001)	0.000003 (0.000001)
*f*_3_	304.359111 (513.738959)	93.636178 (80.553169)	91.3741 (73.55367)
*f*_4_	12.500000 (4.960186)	0.033333 (0.182574)	0.028978 (0.168912)
*f*_5_	4570.725435 (1625.045376)	1841.741864 (711.620590)	1792.6421 (691.28015)
*f*_6_	0 26.074848 (8.945656)	0.000382 (0.000000)	0.000287 (0.000000)
*f*_7_	0.699759 (0.701654)	0.230684 (0.442564)	0.197635 (0.38745)

**Table 2:** Parameter settings of DHSPM for test systems.

HMS	bw	*η*_*m*_	NI
5	0.01	10	50000

**Table 3:** Units data for 3 thermal units' system.

Generator	*P*_min⁡_ (MW)	*P*_max⁡_ (MW)	*a*	*b*	*c*	*e*	*f*
1	100	600	0.001562	7.92	561	300	0.0315
2	50	200	0.00482	7.97	78	150	0.063
3	100	400	0.00194	7.85	310	200	0.042

**Table 4:** 3 thermal units' test results.

Generator	Power (MW)
1	300.12
2	149.88
3	400

**Table 5:** Best result comparison with different algorithms for 3 thermal units' system.

Algorithms	3 thermal units ($) Best result	3 thermal units ($) Average result
CEP [21]	8234.07	8235.97
FEP [21]	8234.07	8234.24
MFEP [21]	8234.08	8234.71
IFEP [21]	8234.07	8234.16
EGA [21]	8234.07	8234.41
FIA [21]	8234.07	8234.26
SPSO [21]	8234.07	8234.18
QPSO [21]	8234.07	8234.10
HS	8234.07	8234.15
IHS	8234.07	8234.13
DHSPM	**8234.07**	**8234.09**

**Table 6:** Units data for 13 thermal units' system.

Generator	*P*_min⁡_ (MW)	*P*_max⁡_ (MW)	*a*	*b*	*c*	*e*	*f*
1	0	680	0.00028	8.1	550	300	0.035
2	0	360	0.00056	8.1	309	200	0.042
3	0	360	0.00056	8.1	307	150	0.042
4	60	180	0.00324	7.74	240	150	0.063
5	60	180	0.00324	7.74	240	150	0.063
6	60	180	0.00324	7.74	240	150	0.063
7	60	180	0.00324	7.74	240	150	0.063
8	60	180	0.00324	7.74	240	150	0.063
9	60	180	0.00324	7.74	240	150	0.063
10	40	120	0.00284	8.6	126	100	0.084
11	40	120	0.00284	8.6	126	100	0.084
12	55	120	0.00284	8.6	126	100	0.084
13	55	120	0.00284	8.6	126	100	0.084

**Table 7:** 13 thermal units' test results.

Generator	Power (MW)
1	628.3205
2	149.6024
3	222.7751
4	109.8655
5	109.8620
6	109.8582
7	60.0008
8	109.8614
9	109.8663
10	39.9997
11	39.9877
12	55.0001
13	55.0003

**Table 8:** Best result comparison with different algorithms for 13 thermal units' system.

Algorithms	13 thermal units ($) Best result	13 thermal units ($) Average result
CEP [21]	18048.21	18190.32
FEP [21]	18018.00	18200.79
MFEP [21]	18028.09	18192.00
IFEP [21]	17994.07	18127.06
EGA [21]	18019.15	18144.95
FIA [21]	18014.61	18136.97
SPSO [21]	17988.15	18102.48
QPSO [21]	17969.01	18075.11
DEC-SQP [7]	17963.94	NR
STHDE [22]	17963.89	NR
IGA_MU [23]	17963.98	NR
SDE [24]	17960.71	NR
HS	17963.91	18065.12
IHS	17962.87	18042.14
DHSPM	**17960.54**	**17994.16**

NR: not reported.

The article "Dynamic Harmony Search with Polynomial Mutation Algorithm for Valve-Point Economic Load Dispatch" was retracted in 2016. Reason: concerns about the peer review.

**Table 9:** Units data for 40 thermal units' system.

Generator	*P*_min⁡_ (MW)	*P*_max⁡_ (MW)	*a*	*b*	*c*	*e*	*f*
1	36	114	0.0069	6.73	94.705	100	0.084
2	36	114	0.0069	6.73	94.705	100	0.084
3	60	120	0.02028	7.07	309.54	100	0.084
4	80	190	0.00942	8.18	369.03	150	0.063
5	47	97	0.0114	5.35	148.89	120	0.077
6	68	140	0.01142	8.05	222.33	100	0.084
7	110	300	0.00357	8.03	287.71	200	0.042
8	135	300	0.00492	6.99	391.98	200	0.042
9	135	300	0.00573	6.6	455.76	200	0.042
10	130	300	0.00605	12.9	722.82	200	0.042
11	94	375	0.00515	12.9	635.2	200	0.042
12	94	375	0.00569	12.8	654.69	200	0.042
13	125	500	0.00421	12.5	913.4	300	0.035
14	125	500	0.00752	8.84	1760.4	300	0.035
15	125	500	0.00708	9.15	1728.3	300	0.035
16	125	500	0.00708	9.15	1728.3	300	0.035
17	220	500	0.00313	7.97	647.85	300	0.035
18	220	500	0.00313	7.95	649.69	300	0.035
19	242	550	0.00313	7.97	647.83	300	0.035
20	242	550	0.00313	7.97	647.81	300	0.035
21	254	550	0.00298	6.63	785.96	300	0.035
22	254	550	0.00298	6.63	785.96	300	0.035
23	254	550	0.00284	6.66	794.53	300	0.035
24	254	550	0.00284	6.66	794.53	300	0.035
25	254	550	0.00277	7.1	801.32	300	0.035
26	254	550	0.00277	7.1	801.32	300	0.035
27	10	150	0.52124	3.33	1055.1	120	0.077
28	10	150	0.52124	3.33	1055.1	120	0.077
29	10	150	0.52124	3.33	1055.1	120	0.077
30	47	97	0.0114	5.35	148.89	120	0.077
31	60	190	0.0016	6.43	222.92	150	0.063
32	60	190	0.0016	6.43	222.92	150	0.063
33	60	190	0.0016	6.43	222.92	150	0.063
34	90	200	0.0001	8.95	107.87	200	0.042
35	90	200	0.0001	8.62	116.58	200	0.042
36	90	200	0.0001	8.62	116.58	200	0.042
37	25	110	0.0161	5.88	307.45	80	0.098
38	25	110	0.0161	5.88	307.45	80	0.098
39	25	110	0.0161	5.88	307.45	80	0.098
40	242	550	0.00313	7.97	647.83	300	0.035

**Table 10:** 40 thermal units' test results.

Generator	Power (MW)
1	110.802
2	110.800
3	97.400
4	179.733
5	87.800
6	140.000
7	259.600
8	284.601
9	284.599
10	130.000
11	94.000
12	94.001
13	214.760
14	394.279
15	394.279
16	394.278
17	489.280
18	489.279
19	511.279
20	511.279
21	523.280
22	523.279
23	523.278
24	523.279
25	523.279
26	523.280
27	10.000
28	10.000
29	10.000
30	87.800
31	189.999
32	190.000
33	190.000
34	164.800
35	199.996
36	194.401
37	110.000
38	110.000
39	110.000
40	511.279

The article "Dynamic Harmony Search with Polynomial Mutation Algorithm for Valve-Point Economic Load Dispatch" was retracted in 2016. Reason: concerns about the peer review.

**Table 11:** Best result comparison with different algorithms for 40 thermal units' system.

Algorithms	40 thermal units ($) Best result	40 thermal units ($) Average result
CEP [21]	123488.29	124793.48
FEP [21]	122679.71	124119.37
MFEP [21]	122647.57	123489.74
IFEP [21]	122624.35	123382.00
EGA [21]	122022.96	122942.66
FIA [21]	121823.80	122662.48
SPSO [21]	121787.39	122474.40
QPSO [21]	121448.21	122225.07
DEC-SQP [7]	121741.97	122295.12
STHDE [22]	121698.51	122304.30
SDE [23]	121412.78	121412.54
HS	121438.24	122221.14
IHS	121435.16	122219.28
DHSPM	**121412.66**	**121423.57**
